The article "Effects of HDM2 antagonism on sunitinib resistance, p53 activation, SDF-1 induction, and tumor infiltration by CD11b+/Gr-1+ myeloid derived suppressor cells" was retracted in 2021. Reasons: fabricated or falsified data; fabricated or falsified images; an official misconduct investigation; misconduct by an author.

# Effects of HDM2 antagonism on sunitinib resistance, p53 activation, SDF-1 induction, and tumor infiltration by CD11b^+^/Gr-1^+^ myeloid derived suppressor cells

**DOI:** 10.1186/1476-4598-12-17

**Published:** 2013-03-05

**Authors:** David J Panka, Qingjun Liu, Andrew K Geissler, James W Mier

**Affiliations:** 1 Division of Hematology-Oncology, Beth Israel Deaconess Medical Center and Harvard Medical School, Boston, MA, USA; 2 Division of Urology, Beijing Friendship Hospital, Capital Medical University, Beijing, China; 3 330 Brookline Avenue, RW-571, Boston, MA, 02215, USA; 4 330 Brookline Avenue, RW-563A, Boston, MA, 02215, USA

**Keywords:** p53, HDM2, HDMX, MI-319, Renal cell carcinoma, Myeloid-derived suppressor cells (MDSC), SDF-1, Endostatin, Collagen prolyl hydroxylase

## Abstract

**Background:**

The studies reported herein were undertaken to determine if the angiostatic function of p53 could be exploited as an adjunct to VEGF-targeted therapy in the treatment of renal cell carcinoma (RCC).

**Methods:**

Nude/beige mice bearing human RCC xenografts were treated with various combinations of sunitinib and the HDM2 antagonist MI-319. Tumors were excised at various time points before and during treatment and analyzed by western blot and IHC for evidence of p53 activation and function.

**Results:**

Sunitinib treatment increased p53 levels in RCC xenografts and transiently induced the expression of p21^waf1^, Noxa, and HDM2, the levels of which subsequently declined to baseline (or undetectable) with the emergence of sunitinib resistance. The development of resistance and the suppression of p53-dependent gene expression temporally correlated with the induction of the p53 antagonist HDMX. The concurrent administration of MI-319 markedly increased the antitumor and anti-angiogenic activities of sunitinib and led to sustained p53-dependent gene expression. It also suppressed the expression of the chemokine SDF-1 (CXCL12) and the influx of CD11b^+^/Gr-1^+^ myeloid-derived suppressor cells (MDSC) otherwise induced by sunitinib. Although p53 knockdown markedly reduced the production of the angiostatic peptide endostatin, the production of endostatin was not augmented by MI-319 treatment.

**Conclusions:**

The evasion of p53 function (possibly through the expression of HDMX) is an essential element in the development of resistance to VEGF-targeted therapy in RCC. The maintenance of p53 function through the concurrent administration of an HDM2 antagonist is an effective means of delaying or preventing the development of resistance.

## Background

One of the major determinants of the response to angiogenesis inhibitors is the p53 status of the tumor cells. Yu *et al*, for example, showed in 2002 that tumors derived from p53^(+/+)^ HCT116 colorectal carcinoma cells were far more sensitive to VEGF receptor targeted therapy than tumors generated from isogenic p53^(-/-)^ cells [1]. This differential sensitivity to treatment correlated with the *in vitro* susceptibility of the tumor cells to the pro-apoptotic effects of hypoxia. Since the publication of these data over a decade ago, the known range of biologic effects regulated by p53 has expanded well beyond cell cycle control and the expression of pro-apoptotic genes to include such diverse functions as the suppression of angiogenesis [2]. It is possible that the differential sensitivity of p53^(-/-)^ and p53^(+/+)^ HCT116 tumors to VEGF receptor-targeted therapy is due to an ability of p53 to complement the effects of VEGF receptor inhibition on the tumor microcirculation.

The article "Effects of HDM2 antagonism on sunitinib resistance, p53 activation, SDF-1 induction, and tumor infiltration by CD11b+/Gr-1+ myeloid derived suppressor cells" was retracted in 2021. Reasons: fabricated or falsified data; fabricated or falsified images; an official misconduct investigation; misconduct by an author.

Although the advent of small molecule inhibitors of VEGFR2 has vastly improved the treatment of patients with renal cell carcinoma (RCC), the response to these agents is generally short-lived [3]. The mechanisms by which tumors ultimately manage to evade the effects of these agents are numerous and only partly understood [3-5]. One such mechanism involves the production of chemokines (e.g. SDF-1, CSF-1, IL-8) that either drive angiogenesis directly or recruit macrophages and other myeloid lineage cells, including CD11b^+^/Gr-1^+^ myeloid-derived suppressor cells (MDSCs), from the bone marrow into tumor tissue [5-11]. These cells produce a variety of factors that promote tumor growth, invasiveness, angiogenesis, and immunosuppression [10-13]. p53 has been shown to suppress the expression of SDF-1 [14,15]. Otherwise, little is known about how the p53 status of a tumor might affect the extent to which tumors are infiltrated by MDSC or the facility with which they develop resistance to VEGF-targeted therapy.

Another mechanism by which p53 suppresses angiogenesis is through the induction of genes that modify the extracellular matrix (ECM). Angiogenesis is negatively regulated, for example, by several ECM-resident peptides (e.g. endostatin, canstatin, arresten) which interact with integrin receptors on the surface of endothelial cells and suppress their proliferation, survival, and motility [16,17]. These peptides are all derived from the noncollagenous (NC1) domains of certain types of collagen through the action of proteases such as MMP9. The genes encoding the collagen α chains (e.g. *COL4A1*) from which these angiostatic peptides are derived as well as that encoding the prolyl hydroxylase needed for the post-translational modification and stabilization of collagen [i.e. α(II) PH] are direct p53 transcriptional targets [18,19]. p53 activation might therefore be expected to suppress the tumor microvasculature through the enhanced production of these peptides. As an illustration of this point, the production of arresten, an angiostatic collagen fragment processed from α1 collagen IV, is markedly diminished in p53^(-/-)^ tumor cells and its overexpression has been shown to retard tumor growth and limit angiogenesis [19]. The role played by these collagen-derived peptides in the regulation of angiogenesis in RCC and the extent to which their production is regulated by p53 is unknown.

p53 levels are generally low in unstressed cells as a result of HDM2-dependent ubiquitination and proteasomal degradation [20]. p53 can be activated as a result of phosphorylation of any of several sites in its N-terminal domain, which dissociates p53 from HDM2 and enhances its stability [21]. Several of the kinases capable of phosphorylating p53 (e.g. ATM) are redox-sensitive and capable of activating p53 in the setting of hypoxia [22]. The p53 gene is intact (i.e. neither deleted, mutated, nor methylated) in most RCC [23]. One might therefore expect p53 to be activated in RCC subjected to the stress of angiogenesis inhibition. Several factors, however, limit the extent, duration, and biological consequences of p53 activation in these cells. RCC, for example, generally fail to express p53-dependent genes in response to DNA damage, presumably due to high constitutive NF-κB activity [24-26]. The transcriptional activity of p53 is also limited by a member of the POK family (KR-POK) frequently overexpressed in RCC [27]. This protein physically interacts with p53 and with the transcriptional corepressors NCoR and BCoR, resulting in reduced histone H3 and H4 acetylation at the promoters of certain p53-dependent genes (e.g. p21^waf1^/CDKN1A). These signaling aberrations suggest that p53 might not be able to contribute to the suppression of angiogenesis or any other biological process in RCC, despite the integrity of the p53 gene. Hammond *et al*, however, have pointed out that many of the functions of p53 in the setting of hypoxia are due to transcriptional repression rather than activation [28-31]. The anti-angiogenic effects of p53, for example, are in part due to the repression of the miR-17-92 microRNA family [32] and possibly to SDF-1 [14,15] and it is unclear how these functions would be affected by constitutive NF-κB activity or KR-POK expression.

The article "Effects of HDM2 antagonism on sunitinib resistance, p53 activation, SDF-1 induction, and tumor infiltration by CD11b+/Gr-1+ myeloid derived suppressor cells" was retracted in 2021. Reasons: fabricated or falsified data; fabricated or falsified images; an official misconduct investigation; misconduct by an author.

Several drugs that inhibit HDM2 are in preclinical or Phase I trials [33-35]. These drugs offer distinct advantages over conventional chemotherapy in that they are able to activate p53 in genetically permissive tumor cells without inducing DNA damage. The studies described in this paper were undertaken to assess the effects of HDM2 blockade alone and in conjunction with VEGF-targeted therapies on p53 function, tumor growth, and angiogenesis in RCC.

## Results

### Sunitinib-induced p53 activation in RCC xenografts

To assess the effects of sunitinib treatment on tumor cell p53 levels and transcriptional activity, 1 × 10^7^ 786-0 or A498 cells were implanted subcutaneously into the flanks of nude/beige mice and the resulting tumors allowed to grow to a diameter of 10 mm, at which point sunitinib treatment (50 mg/kg daily) was begun. The growth of 786-0 xenografts is typically arrested by sunitinib for a period of only 7-10 days, after which growth resumes despite the continued administration of the drug [36]. In the case of A498 xenografts, sunitinib-induced growth arrest extends to approximately 40 days, after which the tumors become resistant to treatment. With each xenograft model, the tumor-bearing mice were randomly divided into three groups and sacrificed at one of three time points, after which the tumors were promptly excised and frozen in liquid N_2_. One-third of the tumor-bearing mice were untreated and sacrificed when the tumors reached 16 mm in diameter. Half of the remaining mice were sacrificed at a point when tumor measurements were stable on treatment (day 3), and the other half were sacrificed at a point when sunitinib resistance had developed (tumor size 16 mm).

Tumors were thawed, lysed, and the lysates analyzed by western blot for p53, and the p53 dependent genes p21^waf1^, HDM2, HDMX, and NOXA. As shown in Figure 1, p53 levels increased markedly in response to sunitinib administration and remained elevated throughout the course of treatment in both 786-0 and A498 xenografts. The p53-dependent genes encoding p21^waf1^ and HDM2 were also induced early during treatment but this effect was transient in that the levels of both proteins reverted to baseline with the emergence of drug resistance, despite persistent expression of p53. NOXA was undetectable in untreated 786-0 and minimally expressed in A498 xenografts. However, in both xenografts, levels rose significantly early during treatment only to decline with the development of resistance. The p53 antagonist HDMX was also constitutively present in A498 and 786-0 xenografts and in both models, HDMX disappeared from the tumor lysates early during treatment only to reappear with the development of resistance. These data suggest that although p53 is stably induced by sunitinib treatment, its function as a transcription factor becomes impaired at some time point during treatment. The data also establish a temporal link between this loss of p53 function, the induction of HDMX, and the development of sunitinib resistance.

The article "Effects of HDM2 antagonism on sunitinib resistance, p53 activation, SDF-1 induction, and tumor infiltration by CD11b+/Gr-1+ myeloid derived suppressor cells" was retracted in 2021. Reasons: fabricated or falsified data; fabricated or falsified images; an official misconduct investigation; misconduct by an author.

**Figure 1:** **p53 activation in 786-0 and A498 RCC xenografts during sunitinib treatment.** Lysates were from control (vehicle only), sunitinib, day 3 (sunitinib responding) and sunitinib, day 21 (suntinib resistant) mice. Lanes represent data from individual tumors for each treatment group. Blots were probed for p53, and the p53 dependent genes noxa, hdm2 and p21, as well as hdmx and vinculin.

### Effect of HDM2/HDMX inhibition on tumor growth and p53 function

To assess the effect of HDM2/HDMX inhibition on tumor growth, 786-0 and A498 tumors generated as described above and in Methods were allowed to reach a diameter of 10 mm. Tumor-bearing mice were then divided into four treatment groups and treated with either sunitinib (50 mg/kg), the HDM2/HDMX antagonist MI-319 (200 mg/kg), both drugs, or saline daily by gavage. As shown in Figure 2A, sunitinib and MI-319 had only a modest growth-retarding effect on 786-0 xenografts when the drugs were administered individually. However, the combination of both drugs actually induced tumor regression (p < 0.0001 combination vs suntinib alone; p < 0.0002 vs MI-319 alone). Sunitinib as a single agent had a more pronounced effect on A498 than on 786-0 xenografts. MI-319 likewise had single agent activity in this model and augmented that of sunitinib (p < 0.006 combination vs suntinib alone; p < 0.0187 vs MI-319 alone). The basis for the different responses of these two VHL-deficient RCC cell lines to treatment is unknown.

**Figure 2:** **A). Effects of sunitinib and MI-319 on the growth of 786-0 and A498 xenografts.** Tumor volume was normalized to the initial volume when treatment began for each individual tumor for each treatment group. Each growth curve represents the mean from 6 mice in each treatment group. **B**). p53 activation in RCC xenografts. Lysates were from tumors on day 21 after the start of treatment. Lanes represent data from individual tumors for each treatment group. Blots were probed for p53, and the p53 dependent genes hdm2 and p21, as well as hdmx and vinculin.

In this study, all tumors were removed on day 21 or when the untreated tumors reached a diameter of 20 mm. Excised tumors were then divided and one half frozen for biochemical analysis and the other half paraffin-embedded for IHC. As shown in Figure 2B, p21^waf1^ was undetectable in the 786-0 tumors from sunitinib alone-treated mice (despite abundant p53) but readily seen in the tumors from the dually treated xenografts. HDM2 was detectable in the tumors from mice treated with MI-319 alone or the drug combination, but not in those from mice that received sunitinib alone. In the A498 xenografts, both p21^waf1^ and HDM2 were absent from the sunitinib alone-treated tumors but abundant in the tumors excised from mice treated with either MI-319 alone or the sunitinib/MI-319 combination. HDMX was present in all tumors except those from the untreated (control) mice. These data indicate that the concurrent administration of MI-319 is able to maintain the expression of the p53-dependent genes p21^waf1^ and HDM2 despite the presence of HDMX, suggesting that MI-319 has significant activity against both HDM2 and HDMX.

The article "Effects of HDM2 antagonism on sunitinib resistance, p53 activation, SDF-1 induction, and tumor infiltration by CD11b+/Gr-1+ myeloid derived suppressor cells" was retracted in 2021. Reasons: fabricated or falsified data; fabricated or falsified images; an official misconduct investigation; misconduct by an author.

### Proapoptotic, antiproliferative and antiangiogenic effects of MI-319

To assess the ability of MI-319 and sunitinib treatment to induce tumor cell apoptosis, TUNEL assays were performed on histologic sections of tumors obtained from mice in the various treatment groups. Sunitinib (but not MI-319) treatment resulted in a significant increase in the number of TUNEL-positive cells in both tumor models (p < .001 vs control for both 786-0 and A498) However, MI-319 increased the pro-apoptotic effect of sunitinib only in 786-0 (p <0.021), but not A498 xenografts (Figure 3A).

**Figure 3:** **Effects of treatment on (A and B) apoptosis (tunel) and (C and D) proliferation in RCC xenografts.** In both 786-0 (**A**) and A498 (**B**) models, sunitinib induced apoptosis as shown by an increase in tunel positive cells. The addition of MI-319 increased apoptosis in 786-0 but not A498 xenografts. Data is presented as a bar graph showing the mean percent tunel positive cells from six tumors in each treatment group. Sunitinib treatment increased Ki-67 nuclear staining in 786-0 (**C**) but not A498 (**D**) xenografts. The Ki-67 staining in 786-0 xenografts from suntinib treatment was suppressed in the presence of MI-319. Data is presented as a bar graph showing the mean percent Ki-67 positive cells from six tumors in each treatment group.

The effects of the two drugs on proliferation were assessed by Ki-67 staining. Sunitinib treatment increased the number of cycling cells only in 786-0 xenografts (p < 0.05) and this proliferative effect was blocked by MI-319 (p < 0.004). As a single agent, MI-319 had no discernible antiproliferative effect in either 786-0 or A498 xenografts (Figure 3B).

The antiangiogenic effects of sunitinib and MI-319 were assessed by IHC using an anti-CD31 antibody. As shown in Figure 4, both drugs individually induced a marked decline in microvessel density (MVD) (p < 0.0001 for either drug vs untreated) in both xenograft models and in 786-0 xenografts, the effects of the two drugs were additive (p < 0.0007 for both drugs vs sunitinib).

The article "Effects of HDM2 antagonism on sunitinib resistance, p53 activation, SDF-1 induction, and tumor infiltration by CD11b+/Gr-1+ myeloid derived suppressor cells" was retracted in 2021. Reasons: fabricated or falsified data; fabricated or falsified images; an official misconduct investigation; misconduct by an author.

**Figure 4:** **Effects of treatment on microvessel density (MVD) in RCC xenografts.** In both (**A**) 786-0 and (**B**) A498 models, sunitinib and MI-319 suppressed tumor angiogenesis. In 786-0, the effects of the two drugs were additive. Data is presented as a bar graph showing the mean MVD from six tumors in each treatment group. A representative tumor section stained for CD31 from each treatment group for 786-0 and A498 xenografts are in **C** and **D**, respectively.

### Effect of MI-319 on sunitinib-induced tumor infiltration by CD11b^+^/Gr-1^+^ MDSC

Tumor-infiltrating myeloid-derived suppressor cells (MDSC) dually expressing CD11b and Gr-1 have been shown to contribute to the development of resistance to several forms of treatment, including antiangiogenic agents that target VEGF receptor signaling [5-11]. To assess the effects of sunitinib and MI-319 on the accumulation of these cells in tumor tissue, tumors of mice from the various treatment groups were analyzed by immunofluorescence. Photographs of the 786-0 slides are shown in Figure 5A and bar graphs of the data from both 786-0 and A498 tumors are shown in Figure 5B. As shown in the figure, very few CD11b^+^/Gr-1^+^ MDSC were detected in untreated 786-0 or A498 xenografts. However, in both xenografts, sunitinib treatment induced an influx of these cells (p < 0.0001 for 786-0, sunitinib vs untreated; p < 0.021 for A498) which was markedly attenuated by the concurrent administration of MI-319 (p < 0.0001 for 786-0, both drugs vs sunitinib; p < 0.036 for A498). In the 786-0 model, this suppression of MDSC tumor infiltration was essentially complete. Of note, MI-319 did not suppress tumor infiltration by all myeloid cells as indicated by the persistence of red (but not magenta) cells in the dually treated tumors. The total number of CD11b^+^ cells present within the tumors was essentially the same in the sunitinib and sunitinib/MI-319 treatment groups, suggesting that the suppressive effects of MI-319 were directed at specific subpopulations of CD11b^+^ myeloid cells.

**Figure 5:** **Effects of treatment on CD11b**^**+/**^**Gr-1**^**+ **^**MDSC infiltration into 786-0 and A498 xenografts. A**). Immunofluoresence data from 786-0 xenografts. In this study, CD11b = red, Gr-1 = blue. Dually expressing cells are magenta colored; tumor nuclei are yellow. **B**). Bar graph generated from the manual counting of CD11b^+/^Gr-1^+^ cells from five individual tumors from each treatment group. Data from both 786-0 and A498 xenografts are shown. **C**). SDF-1 levels in RCC xenografts. Lysates were from tumors on day 21 after the start of treatment. Lanes represent data from individual tumors for each treatment group.

The article "Effects of HDM2 antagonism on sunitinib resistance, p53 activation, SDF-1 induction, and tumor infiltration by CD11b+/Gr-1+ myeloid derived suppressor cells" was retracted in 2021. Reasons: fabricated or falsified data; fabricated or falsified images; an official misconduct investigation; misconduct by an author.

The accumulation of CD11b^+^/Gr-1^+^ MDSC within tumor tissue is driven by several chemokines (e.g. SDF-1) produced by tumor and associated stromal cells [5-11]. The production of the SDF-1 is known to be hypoxia-induced and negatively regulated by p53 [14,15]. One would therefore predict that treatment with an angiogenesis inhibitor such as sunitinib would induce the expression of SDF-1 and the concurrent administration of an HDM2 antagonist such as MI-319 might block this induction. To test this hypothesis, tumor lysates from the various treatment groups were analyzed by western blot for SDF-1. As shown in Figure 5C, SDF-1 was not detected in 786-0 tumor lysates from untreated mice. Sunitinib treatment induced SDF-1 expression, however, and this induction was completely suppressed by the concurrent administration of MI-319. In A498 xenografts, SDF-1 was present constitutively but increased with sunitinib treatment. As with the 786-0 xenografts, this induction was suppressed by MI-319.

### α(II) prolyl hydroxylase induction by sunitinib: effects of treatment on endostatin and arresten deposition

α(II) PH is essential for the proper post-translational modification and stabilization of collagen α chains and for the production of angiostatic peptides (e.g. endostatin, canstatin, arresten) from their non-collagenous NC1 domains [18,19]. The gene encoding this enzyme is p53-dependent. To determine the extent to which p53 activation regulates the deposition of endostatin and arresten in the ECM of RCC, mice bearing xenografts generated from 786-0 stably transfected with a tetracycline-regulable p53 shRNA (see Methods) were treated with sunitinib with or without the inclusion of doxycycline in the drinking water. The mice were then sacrificed and the tumors excised. As shown in Figure 6A, sunitinib treatment was less effective in the absence of p53, especially during the first few days of treatment (p < 0.025 at day 7, sunitinib alone vs sunitinib + doxycycline). In fact, the growth curve of the sunitinib + doxycycline-treated mice overlapped with that of the control mice. Analysis of tumor lysates showed a complete suppression of endostatin and arresten production by the tumors that failed to activate p53 in response to sunitinib (Figure 6B). These data suggest that p53 activation is essential for the deposition of endostatin and arresten triggered by the administration of sunitinib in RCC xenografts.

**Figure 6:** **A). Effect of p53 knockdown on the response of 786-0 xenografts to sunitinib treatment.** The expression of a p53 shRNA markedly reduced the antitumor effect of sunitinib. Each growth curve represents the mean tumor volume from 6 mice in each treatment group. **B**). p53 knockdown blocked the deposition of endostatin and arresten otherwise induced by sunitinib treatment. Lysates were from tumors on day 28 after the start of treatment. Lanes represent data from individual tumors for each treatment group. Blots were probed for p53, p21, endostatin, arresten and vinculin.

The article "Effects of HDM2 antagonism on sunitinib resistance, p53 activation, SDF-1 induction, and tumor infiltration by CD11b+/Gr-1+ myeloid derived suppressor cells" was retracted in 2021. Reasons: fabricated or falsified data; fabricated or falsified images; an official misconduct investigation; misconduct by an author.

To determine if the variable p53 function observed during the course of treatment with sunitinib affected the levels of α(II) PH, endostatin and arresten, the tumor lysates from Figure 1 were analyzed by western blot for these proteins. As shown in Figure 7A and B, low levels of α(II) PH, endostatin and arresten were detectable in untreated 786-0 and A498 xenografts, but all three proteins were up regulated by sunitinib treatment. However, in contrast to p21, Noxa, and HDM2, which nearly disappeared with the development of resistance (Figure 1), endostatin and arresten persisted at nearly the same level with the onset of drug resistance. These data suggest that sustained p53 transcriptional activity is not required to maintain endostatin and arresten levels in the tumor ECM and that the development of resistance cannot be due to a reduction in the level of these angiostatic peptides.

**Figure 7:** **The effects of treatment on α(II) PH, endostatin, and arresten levels in RCC xenografts. A, B**). The expression of all three proteins was induced by sunitinib treatment and levels did not diminish with the onset of drug resistance. **C**, **D**). Levels of endostatin and arresten were increased by treatment with either sunitinib or MI-319 but the inductive effects of the two drugs were not additive. Lanes represent data from individual tumors for each treatment group.

To determine if HDM2 blockade could increase endostatin or arresten levels beyond those achieved with sunitinib alone, 786-0 xenografts were treated with sunitinib, MI-319, or both drugs and the tumors examined by western blot. As shown in Figure 7C and D, the levels of neither endostatin nor arresten were further increased by the concurrent administration of MI-319 in either 786-0 or A498 xenografts. These data suggest that the transient activation of p53 induced by sunitinib treatment in genetically permissive RCC is sufficient to maximize the deposition of endostatin and arresten in the ECM. The data also suggest that the superior antitumor and anti-angiogenic effects of the sunitinib/MI-319 combination cannot be explained by an increase in the abundance of these angiostatic collagen fragments in the ECM. Of note, single agent MI-319 increased p21^waf1^ and arresten levels in A498 xenografts, the only model of the two evaluated in which the drug had single agent antitumor activity.

The article "Effects of HDM2 antagonism on sunitinib resistance, p53 activation, SDF-1 induction, and tumor infiltration by CD11b+/Gr-1+ myeloid derived suppressor cells" was retracted in 2021. Reasons: fabricated or falsified data; fabricated or falsified images; an official misconduct investigation; misconduct by an author.

## Discussion

Despite the numerous constraints on p53 function in RCC [24-27], sunitinib treatment does induce the expression of several p53-dependent genes (e.g. NOXA, HDM2, p21^waf^) in RCC xenografts. The induction of these genes is, however, limited to the interval during which tumor growth is suppressed and is attenuated once resistance develops. Although several factors have been shown to block p53 transcriptional activity in RCC, these are for the most part stable genetic alterations (e.g. KR-POK expression) that are not known to be subject to regulation by hypoxia or other metabolic changes that occur during treatment with angiogenesis inhibitors.

The factor(s) responsible for the transient activation and subsequent inactivation of p53 transcriptional activity during the course of treatment with sunitinib are unknown but at least one well-characterized p53 transcriptional suppressant (i.e. HDMX) appears to be temporally linked to p53 function in our xenograft models and may therefore be a candidate. Unlike its binding partner HDM2, HDMX is not regulated by p53 [37]. HDMX is constitutively expressed in RCC xenografts but vanishes with the initiation of sunitinib treatment – along with the appearance of p21^waf^. HDMX reappears with the development of resistance, in association with the down modulation of p21^waf^. These temporal associations strongly implicate HDMX as the factor responsible for the failure of p53 to maintain p21^waf1^ expression. The reappearance of HDMX during sunitinib treatment also explains why the suppression of p53 with an shRNA affected the response of 786-0 xenografts to sunitinib only during the first few days of treatment. As shown in Figure 6A, the xenografts in which p53 activation is not impeded characteristically stall for several days during sunitinib treatment but subsequently catch up with those in which p53 expression is suppressed. These data are consistent with the inactivation of p53 function by HDMX.

HDMX is physically associated with HDM2 and drugs that block the interaction between HDM2 and p53 such as MI-319 also interfere to some extent with the ability of HDMX to suppress p53 transcriptional activity. The fact that MI-319 maintains p21^waf^ levels during sunitinib treatment suggests that the factor responsible for limiting p53 nuclear function most likely interacts with HDM2. This consideration, in addition to the temporal linkage between HDMX expression and the absence of p21^waf^, supports the hypothesis that HDMX is the dominant regulator of p53 nuclear function during sunitinib treatment and possibly a major factor in the development of drug resistance.

The article "Effects of HDM2 antagonism on sunitinib resistance, p53 activation, SDF-1 induction, and tumor infiltration by CD11b+/Gr-1+ myeloid derived suppressor cells" was retracted in 2021. Reasons: fabricated or falsified data; fabricated or falsified images; an official misconduct investigation; misconduct by an author.

Despite the induction of p21 (Figure 2B), MI-319 treatment does not have a consistent effect on tumor cell proliferation as determined by Ki67 staining (Figure 3). In A498 xenografts, for example, MI-319 neither retards proliferation when administered as a single agent or when given concurrently with sunitinib. In 786-0 xenografts, however, the addition of MI-319 suppresses the increase in proliferation induced by sunitinib treatment. The enhanced tumor cell proliferation induced by sunitinib is presumably the result of tumor hypoxia, which has been reported to enhance proliferation in other tumor models [38].

The anti-angiogenic effect of sunitinib is augmented by the concurrent administration of MI-319. One mechanism by which MI-319 might further limit angiogenesis is the suppression of the influx of MDSC that generally occurs in response to sunitinib treatment. This suppressive effect is particularly obvious in 786-0 xenografts, from which MDSC are virtually excluded by MI-319 treatment. The means by which MI-319 (and p53) inhibit MDSC trafficking from the bone marrow to tumor tissue is not known but may involve the suppression of chemokine (e.g. SDF-1) production by tumor cells and stromal elements that were rendered hypoxic by the disruption of the tumor vasculature. The ability of MI-319 to suppress both baseline and sunitinib-induced SDF-1 expression in our RCC xenografts is consistent with the known ability of p53 to suppress SDF-1 expression [14,15]. Although our data suggest that the suppression of SDF-1 may account for the diminution in the influx of MDSC observed in the tumor infiltrates of mice treated with MI-319, it is possible that other factors that are both hypoxia-inducible and suppressed by p53 will be identified that might contribute to the anti-angiogenic effects of the drug.

Our observation that sunitinib treatment increases MDSC infiltration of RCC xenografts is at odds with several previous reports showing that the drug limits the expansion of these cells and enhances immune function [39-43]. Most of these earlier reports, however, were based on analyses of peripheral blood or splenocytes. Ko *et al*, for example, showed that RCC patients have increased numbers of MDSC in the peripheral blood and that sunitinib treatment results in a decline in their numbers [39]. Sunitinib treatment consistently reduces MDSC accumulation in the spleens of tumor-bearing mice in several tumor models [40]. However, this effect on splenic MDSC did not extend to the tumor microenvironment, where MDSC continued to accumulate with the expected deleterious effect on T cell function, regardless of treatment. These site-specific effects may be attributable to the cytokine GM-CSF, which is capable of rendering MDSC resistant to the effects of sunitinib [40].

The article "Effects of HDM2 antagonism on sunitinib resistance, p53 activation, SDF-1 induction, and tumor infiltration by CD11b+/Gr-1+ myeloid derived suppressor cells" was retracted in 2021. Reasons: fabricated or falsified data; fabricated or falsified images; an official misconduct investigation; misconduct by an author.

Our studies suggest that sunitinib can actually increase the influx of MDSC into tumor tissue in some circumstances. This result may be unique to VHL-deficient RCC and dependent on the severity of the hypoxia induced in these tumors by VEGF-targeted agents. To the extent that this is the case, one would expect that these tumors would abundantly produce SDF-1 and other HIF-dependent chemokines (which recruit MDSC) in response to sunitinib treatment. The suppressive effects of sunitinib on MDSC accumulation and function are thought to be mediated through the inhibition of STAT3 and c-kit [41,42]. It is possible that hypoxia-induced chemokine production within tumor tissue may in some circumstances trump these inhibitory effects of sunitinib, resulting in an increase in MDSC infiltration.

Another mechanism by which p53 regulates angiogenesis is through the induction of α(II) PH and the deposition of anti-angiogenic collagen fragments (e.g. arresten, endostatin, canstatin) in the ECM [16-19]. Several previous studies have in fact suggested that this is one of the dominant mechanisms by which tumor angiogenesis and growth are suppressed by p53 [19]. Our data clearly establish that p53 activation is essential for the deposition of endostatin and arresten in 786-0 xenografts (Figure 6A) and in this respect, our results corroborate the results of Assadian *et al*, who demonstrated a similar requirement for p53 in the production of arresten by HCT116 cells [19]. Despite the absolute requirement for p53, however, sustained p53 activation does not appear to be essential to maintain endostatin and arresten levels in RCC xenografts during sunitinib treatment. We have not been able to demonstrate a significant decline in endostatin or arresten levels after the initial induction despite the apparent loss of p53 transcriptional activity (i.e. the disappearance of p21^waf1^) during treatment. Indeed, endostatin and arresten levels remain nearly unchanged with the development of sunitinib resistance, when p21^waf1^ is no longer detectable. Nor have we been able to demonstrate any enhancement in endostatin or arresten deposition by the addition of MI-319 to the treatment regimen, although HDM2 antagonism is essential for the maintenance of p21^waf1^ expression. Collectively, these data suggest that although the failure to express α(II) PH and to deposit angiostatic collagen fragments (e.g. endostatin, arresten) in the ECM might account for the faster growth and more vigorous angiogenesis observed in p53^(-/-)^ tumors, changes in endostatin or arresten levels are not a factor in the development of sunitinib resistance in p53-WT RCC nor in the enhanced suppression of angiogenesis and tumor growth resulting from the concurrent administration of MI-319 with sunitinib.

The article "Effects of HDM2 antagonism on sunitinib resistance, p53 activation, SDF-1 induction, and tumor infiltration by CD11b+/Gr-1+ myeloid derived suppressor cells" was retracted in 2021. Reasons: fabricated or falsified data; fabricated or falsified images; an official misconduct investigation; misconduct by an author.

We have demonstrated that treatment of mice bearing RCC xenografts with VEGF-targeted agents results in p53 activation, the biological effects of which are quickly undermined with the onset of drug resistance, possibly due to the induction of the p53 antagonist HDMX. We have further shown that the HDM2/HDMX antagonist MI-319 maintains p53 function during treatment and delays/prevents the emergence of resistance. These data suggest that the evasion of p53 function is an essential element in tumor escape from the effects of VEGF-targeted therapy. The effects of MI-319 appear to be at least in part due to the ability of the drug to suppress the influx of MDSC into the tumor, which may in turn be due to its ability to block the production of chemokines such as SDF-1 that are otherwise induced in the setting of hypoxia. The potential utility of a combination of an HDM2 antagonist with sunitinib may not be limited to RCC. For example, in a recent study by Henze *et al*, the HDM2 antagonist Nutlin-3 was shown to augment the apoptotic response of imatinib-resistant gastrointestinal stromal tumor (GIST) cell lines to sunitinib [44]. In this case, however, the effects of sunitinib were most likely attributable to its ability to inhibit c-kit rather than its antiangiogenic effects. Collectively, these data provide a strong rationale for the concurrent use of HDM2 antagonists as adjuncts to VEGF receptor inhibitors in the management of metastatic RCC and other tumor types.

## Materials and methods

Cell lines and reagents. The human RCC cell lines 786-0 and A498 were obtained from ATCC and maintained in RPMI-1640 (Lonza) and Eagle minimal essential medium (ATCC), respectively containing 10% fetal bovine serum (USA Scientific), 2 mM glutamine and 50 μg/ml gentamycin at 37°C in 5 percent CO_2_. The MI-319 was provided by Ascenta Therapeutics (Malvern, PA) and Sanofi-Aventis (Paris, France).

### Western blots

Cells were treated as described in Results and then lysed in Lysis Solution (Cell Signaling) supplemented with sodium fluoride (10 μM, Fisher Scientific, Hampton, NH) and phenylmethylsulfonyl fluoride (100 μg/ml, Sigma-Aldrich, St Louis, MO). Lysates were fractionated in 8-16% gradient SDS-polyacrylamide gels as indicated and the separated proteins were transferred to nitrocellulose. The blots were probed for the proteins of interest with specific antibodies followed by a second antibody-horse radish peroxidase conjugate and then incubated with SuperSignal chemiluminescence substrate (Pierce, Rochford, IL). The blots were then exposed to Kodak X-Omat Blue XB-1 film. The p21^waf1^, noxa, SDF-1, collagen type XVIII (endostatin) and collagen type IV (arresten) antibodies were obtained from Santa Cruz Biotechnology (Santa Cruz, CA); the p53 antibody was purchased from Cell Signaling (Beverly, MA); the HDMX and HDM2 antibodies were obtained from ABCAM (Cambridge, MA). The vinculin antibody was obtained from Sigma (St. Louis, MO). The CD11b antibody conjugated to Alexa 488 and the Gr-1 antibody conjugated to Alexa 647 were purchased from Biolegend (San Diego, CA). The α(II) PH antibody was obtained from Bethyl Laboratories (Montgomery, TX).

The article "Effects of HDM2 antagonism on sunitinib resistance, p53 activation, SDF-1 induction, and tumor infiltration by CD11b+/Gr-1+ myeloid derived suppressor cells" was retracted in 2021. Reasons: fabricated or falsified data; fabricated or falsified images; an official misconduct investigation; misconduct by an author.

### Xenograft model

All animal studies were conducted according to an Institutional Animal Care and Use Committee (IACUC)-approved protocol at the Beth Israel Deaconess Medical Center. Six to eight week old athymic nude/beige female mice (Charles River Labs) were implanted subcutaneously with 1.0 × 10^7^ RCC cells. When the tumors reached 10 mm in diameter, the mice were divided into 4 treatment groups of 6 mice each and treated daily for 21 days by gavage with sunitinib (50 mg/kg), MI-319 (200 mg/kg), sunitinib + MI-319, or saline (control). The doses of sunitinib [36,45] and MI-319 [46,47] were as previously reported. Tumors were measured bidimensionally daily. Tumor tissue from the sacrificed mice was frozen in liquid N_2_ for western blot analysis as described in Results or fixed in formalin for paraffin embedding.

### Immunohistochemistry and immunofluorescence microscopy

The paraffin-embedded tumor tissue was sectioned at 5 microns using a Leica RM 2125 rotary microtome. The sections were dewaxed at 60°C, serially immersed in solutions of decreasing alcohol concentration, and then boiled in 10 mM sodium citrate, pH 6.2, for 30 minutes to unmask antigens. The tissue was then incubated in 3% hydrogen peroxide for 5 minutes, blocked with 1% BSA and 5% goat serum, and incubated overnight at 4°C with an antibody to Ki-67 (Dako, Carpinteria, CA). The Ki-67 epitope was detected using a biotinylated anti-mouse Ig antibody and an avidin-horseradish peroxidase conjugate (Vector Laboratories, Burlingame, CA). Similarly, sections were stained for endothelial cells with an antibody to CD 31 (ABCAM), followed by a biotinylated anti-rabbit Ig antibody (Vector Laboratories, Burlingame, CA). Slides were then counterstained with hematoxylin, dehydrated, and mounted. Tissue staining was quantitated using IMAGE Pro 6.0 software (MediaCybernetics, Inc, Bethesda, MD).

The sections were assayed for apoptosis using the TUNEL method (Millipore, Billerica, MA) in accordance with an established protocol [48]. The tissue was hydrated and treated sequentially with proteinase K and hydrogen peroxide, and then blocked as described above for the Ki-67 staining. The sections were then exposed to a solution containing mixed nucleotides, some of which were digoxygenin-labeled, and terminal deoxynucleotidyl transferase (TdT). The slides were developed with an anti-digoxigenin antibody-peroxidase conjugate and DAB substrate.

The article "Effects of HDM2 antagonism on sunitinib resistance, p53 activation, SDF-1 induction, and tumor infiltration by CD11b+/Gr-1+ myeloid derived suppressor cells" was retracted in 2021. Reasons: fabricated or falsified data; fabricated or falsified images; an official misconduct investigation; misconduct by an author.

Immunofluorescence microscopy was utilized to image the infiltration of the CD11b^+^/ Gr-1^+^ MDSC cells with each paraffin embedded tissue. The protocol followed the procedure outlined above for Ki-67 and CD31 staining for dehydration to hydration and unmasking followed by blocking with 5% normal goat serum in PBS/0.05% triton ×-100. Antibodies to CD11b antibody conjugated to Alexa 488 and the Gr-1 antibody conjugated to Alexa 647 were added concurrently at 1:200 dilution in PBS/1% BSA/0.05% triton ×-100 and incubated overnight at 4°C. After several washings with PBS, nuclei were stained with Bisbenzimide H33342 (Alexis Biochemicals, San Diego, CA). Immunofluoresence microscopy was carried out with a Nikon TE-2000E microscope at 20× magnification and a Hamamatsu Orca ER camera. The data was acquired with Nikon’s NIS-Elements and analyzed with ImageJ software.

### Design and construction of tet-inducible p53 shRNA-transfected 786-0 cell line

To generate 786-0 cells expressing a tetracycline inducible shRNA to p53, the shRNA sequence selector and shRNA hairpin oligonucleotide sequence designer software provided by BD Clontech was used to select optimal sequences. Three shRNAs were generated for each gene to be silenced. To produce tetracycline-regulable shRNAs, the oligonucleotides selected were cloned into the pSingle-tTS-shRNA vector (BD Clontech). This vector is a tet-on vector. The three shRNA constructs were transfected as a group into 786-0 cells and stable transfectants obtained by selection in G418. Clones were screened individually for inducible expression of the shRNA (i.e. the suppression of doxorubicin-induced p53 expression as determined by Western blot) and 2-3 representative clones were selected for each shRNA based on the degree to which tetracycline exposure suppressed p53 expression.

### Statistical analysis

*In vitro* data depicted as bar graphs represent mean values from at least 3 separate experiments +/- standard error. For most of the studies shown, the significance of an apparent difference in mean values for any parameter (e.g. the percent of cells staining with propidium iodide) was validated by a Student’s unpaired *t* test and the difference considered significant if p <0.05. For the xenograft studies, the growth curves of the different treatment groups were statistically compared using one-way ANOVA.

The article "Effects of HDM2 antagonism on sunitinib resistance, p53 activation, SDF-1 induction, and tumor infiltration by CD11b+/Gr-1+ myeloid derived suppressor cells" was retracted in 2021. Reasons: fabricated or falsified data; fabricated or falsified images; an official misconduct investigation; misconduct by an author.

## Abbreviations

SDF-1: Stromal cell-dervived factor-1; VEGF: Vascular endothelial growth factor; PH: Prolyl hydroxylase; RCC: Renal cell carcinoma; ECM: Extracellular matrix; ATM: Ataxia telangiectasia mutated; HDM2: Human double minute 2.

## Competing interests

The authors declare that they have no competing interests.

## Authors’ contributions

QL and AG carried out many of the xenograft experiments, immnuohistochemistry, wide field fluorescence and western blots. JM conceived of the study, and participated in its design and coordination and helped to draft the manuscript. DP also conceived of the study, and participated in its design and coordination and helped to draft the manuscript. In addition, DP performed all in vitro experiments including the generation of tet-regulable shRNA cell lines and their implementation, immnuohistochemistry, wide field fluorescence and western blots. All authors read and approved the final manuscript.
